# DiaMole: Mole Detection and Segmentation Software for Mobile Phone Skin Images

**DOI:** 10.1155/2021/6698176

**Published:** 2021-06-02

**Authors:** Shuai Liu, Zheng Chen, Huahui Zhou, Kunlin He, Meiyu Duan, Qichen Zheng, Pengcheng Xiong, Lan Huang, Qiong Yu, Guoxiong Su, Fengfeng Zhou

**Affiliations:** ^1^College of Computer Science and Technology and Key Laboratory of Symbolic Computation and Knowledge Engineering of Ministry of Education, Jilin University, Changchun 130012, China; ^2^Department of Epidemiology and Biostatistics, School of Public Health, Jilin University, 1163 Xinmin Street, Changchun 130021, China; ^3^Beijing Dr. of Acne Medical Research Institute, Beijing 100000, China

## Abstract

**Results:**

This study developed mole detection and segmentation software DiaMole using mobile phone images. DiaMole utilized multiple deep learning algorithms for the object detection problem and mole segmentation problem. An object detection algorithm generated a rectangle tightly surrounding a mole in the mobile phone image. Moreover, the segmentation algorithm detected the precise boundary of that mole. Three deep learning algorithms were evaluated for their object detection performance. The popular performance metric mean average precision (mAP) was used to evaluate the algorithms. Among the utilized algorithms, the Faster R-CNN could achieve the best mAP = 0.835, and the integrated algorithm could achieve the mAP = 0.4228. Although the integrated algorithm could not achieve the best mAP, it can avoid the missing of detecting the moles. A popular Unet model was utilized to find the precise mole boundary. Clinical users may annotate the detected moles based on their experiences.

**Conclusions:**

DiaMole is user-friendly software for researchers focusing on skin lesions. DiaMole may automatically detect and segment the moles from the mobile phone skin images. The users may also annotate each candidate mole according to their own experiences. The automatically calculated mole image masks and the annotations may be saved for further investigations.

## 1. Introduction

Skin cancer is a major public health problem, and melanoma accounted for 75% of deaths associated with skin cancers [1]. Screening of all skin cancer types before metastasis may provide the patients with more effective treatment options [2]. Noninvasive dermoscopy is a popular technology to capture high-resolution images of skin lesions [2].

Melanoma detection based on mobile phone images recently caught the dermatologic researchers' attention [3, 4]. However, the existing studies did not demonstrate sufficient detection accuracies, and they may even identify melanomas as normal cases with a high likelihood [3]. The MoleMapper project collected the skin moles captured by the iPhone ResearchKit and released the data for the research community [5]. However, this dataset did not provide the detailed masks of the lesion sites and the disease annotations.

Segmentation and classification were the two tasks for the dermoscopy image-based melanoma prediction study [6]. A dermoscopy image usually zoomed in to the skin mole, and segmentation served as the first task to get the skin mole's precise boundary. Zhang et al. coupled a deep fully convolutional network and a shallow network with textons to automatically detect the skin lesions' detailed segmentations [7]. Fully convolutional residual networks also demonstrated promising performances in segmenting the skin lesions on the dermoscopy images [8]. The second task of lesion classification may utilize deep neural networks [8] or regular classifiers like support vector machines (SVMs) [9].

This study hypothesized that locating the lesion site with a rectangle may improve the mole detection using mobile phone images. This was based on the observation that the skin lesion usually occupied the majority area of a dermoscopy image, and usually there was only one lesion per dermoscopy image. The experienced dermatologist may ensure the high quality of a dermoscopy image. However, all these assumptions may not always be correct for a mobile phone image captured by a nonprofessional user. The software DiaMole was proposed to provide both object detection and segmentation functions using popular algorithms. The user may also annotate the moles using their experiences within the software DiaMole.

## 2. Materials and Methods

### 2.1. Summary of the Datasets Used in This Study

Two datasets were used to evaluate the performances of the proposed software DiaMole. The MoleMapper project generously authorized us to evaluate DiaMole using their mole images captured by the Apple ResearchKit [5]. The project recruited 2,069 participants, who contributed 1,920 demographic surveys, 3,274 mole measurements, and 2,422 curated mole images. Each image is 320 × 568 pixels in size. But the current version of the dataset did not provide the annotations of the bounding boxes and mole masks. This study annotated the bounding boxes of the MoleMapper images using the open-source software labelImg [10]. Most of the images in this dataset put coins as the size meters of the moles. This study only keeps the images with both moles and coins for further analysis. There are 2,415 images reserved to train and evaluate our models. We use 70% of the dataset to train our models and 30% to test the trained models. There are 1,691 and 724 images in the training and testing datasets, respectively.

Another public dataset from the ISIC 2018 challenge was retrieved to train our segmentation model [11, 12]. This dataset provides 2,594 images, and each is 224 × 224 pixels in size.

This study was approved by the institutional review board (IRB) of the College of Public Health of the Jilin University. All the recruited local participants signed the informed consent forms. Ten local participants were recruited to collect the mole images captured by mobile phones. There are five male and five female participants in this local cohort. Seven mole images were captured by iPhone 6S, and the operating system is IOS 12.3.1. Each image is 1080 × 1440 pixels in size. To verify the influence by different mobile operating systems, we chose three local participants to collect the mole images by three different mobile operating systems. In this study, we use iPhone XR to collect the images, and the operating system is IOS 14.2, and each image is 4032 × 3024. We use HLK-AL00, and the operating system is Android 10.1.0, and each image is 3000 × 4000. We use OPPO Find X2, and the operating system is Android 10, and each image is 3000 × 4000. This dataset serves as an independent validation and demonstrative dataset for DiaMole. The images of the local cohort were resized to 320 × 568 in pixels, the same size in the MoleMapper cohort.

Although there were over two thousand images in the public datasets, we were concerned about whether the deep learning models could be well trained using these images. So we only split the dataset into 70% training and 30% test datasets. The training dataset was used to train the model and to tune the hyperparameters. The 30% images in the test dataset were not involved in the model training step. This may cause the model overfitting problem. So both the 30% test dataset and the locally collected dataset were used to independently evaluate the trained model. The conventional training/validation/test splitting strategy will be used if a larger dataset is available.

### 2.2. Summary of the DiaMole Implementation

This study developed the mole detection and segmentation software DiaMole using the Python programming language version 3.6.2. Two major Python packages TensorFlow version 1.12.0 and OpenCV version 4.1.1.26 were used to support the object detection and lesion segmentation modules. DiaMole was developed and tested on the two mainstream operating systems Windows 7 and Windows 10.

DiaMole has a few prerequisite Python packages, including Numpy and Pillow. To provide an easy installation procedure, we used the software Anaconda Distribution version 4.3.25 to manage the virtual environments. The virtual environment was exported as the configuration file “diamole.yaml.” The Anaconda Distribution is an open-source Python system that supports Linux, Windows, and Mac OS X. If the user wants to install the running environment, use the command line “conda env create -f diamole.yaml.” Then the environment may be started by the command line “activate diamole.” The graphical user interface (GUI) of DiaMole may be started in the above environment by “python gui\main.py.”

### 2.3. Implementation Details of Object Detection Algorithms

The first main task of DiaMole was object detection, and three popular object detection algorithms were integrated. The popular object detection algorithm YOLOv3 (You Only Look Once) [13] calculated the bounding box of an object at three scales, as similar to the feature pyramid networks [14]. Each bounding box was evaluated using logistic regression, and the class label of each detected box was predicted by a series of 3 × 3 and 1 × 1 convolutional layer duets. YOLOv3 ran very fast to accurately predict the objects and their class labels in the given image.

Another widely used two-stage object detection algorithm, Faster R-CNN (faster region convolutional neural network, abbreviated as FR-CNN), was also integrated into DiaMole [13]. FR-CNN utilized a region proposal network (RPN) to generate high-quality region proposals. Its object detection performance was better than the previous version, the fast region convolutional neural network [15].

Lin et al. proposed RetinaNet, a simple dense detector [16]. RetinaNet matched the running speed of the previous one-stage object detection networks but achieved a better object detection accuracy [16]. The main contribution of RetinaNet was a new focal loss function that reduced the training bias caused by the dataset imbalance and rapidly focused the model training process on the difficult samples.

The detection results of all the above three object detection algorithms might be integrated using the Non-Maximum Suppression (NMS) strategy to generate the consensus object bounding boxes [17]. The integration procedure was denoted as the algorithm ALL.

### 2.4. Implementation Details of Mole Segmentation

The dataset MoleMapper did not provide the mole masks and labels, and this study transferred a publicly available segmentation model from the ISIC 2018 challenge [18]. The ISIC 2018 challenge released a number of segmentation source codes, and the team Opsins released their convolutional neural networks (CNNs) with the UNet architecture. The pretrained VGG-16 model was chosen as the base model in this study [19].

A mole usually occupied the major part of a dermoscopic image, but a mobile phone skin image may cover the large neighboring regions of a few moles. So this study firstly got the bounding boxes of the moles using the above object detection algorithms. Then each bounding box was regarded as a dermoscopy-like image and fed to the segmentation model.

This model was implemented using the Python programming language version 3.6.2. The following Python packages were used in the above-mentioned UNet model: Tensorflow version 1.12.0, Keras version 2.2.4, Pandas version 0.25.1, Numpy version 1.17.2, Scikit-image version 0.16.1, Matplotlib version 3.1.1, etc.

## 3. Results

### 3.1. Workflow of DiaMole

The graphical user interface (GUI) of DiaMole may be loaded by running the command line “python gui/main.py” in the directory of DiaMole, as shown in Figure 1. The default workflow is to detect the moles in a given human skin image. This image may be captured by a mobile phone. The bounding boxes of the moles are detected using the three popular object detection algorithms, that is, YOLOv3, FR-CNN, and RetinaNet. These algorithms' results may also be integrated using the algorithm NMS.

In the second step, the UNet model will get the precise boundary of each mole, whose bounding box is cropped by the detection algorithms. Besides, the user can draw the bounding boxes based on their own experiences for the moles which are not detected by the algorithms. All the annotations could be saved to local database.

All the intermediate data are stored in the local database. The user may export the masks and annotations of the detected moles for further analysis. The user can export the masks, bounding boxes, and annotations of the detected moles to a word file.

### 3.2. Data Analysis and Annotation Protocol Using DiaMole

This section described the data analysis and annotation protocol using the proposed software DiaMole. The experimental data of DiaMole on multiple datasets were described and discussed in the following sections.

  Step 1. Run the software DiaMole and its GUI, as shown in Figure 2(a). The left region consists of two buttons and one text box. The user may click the button “Input an Image” to load one image into DiaMole or click the other button “Choose a Folder” to load all the images into DiaMole. DiaMole can automatically load the images in the specified folder if these images are in the formats of JPG, PNG, BMP, and TIFF.
  The middle region has four buttons, and each is to provide one of the four object detection algorithms, YOLOv3, RetinaNet, FR-CNN, and ALL. The below part is the visualization region, and there are three pages for the raw image (raw), images with bounding boxes (detect), and images for manual curation (draw).
  The right region has three buttons, that is, “About,” “Export,” and “Save.” The button “About” gives a pop-up window with the information about DiaMole. The button “Save” is to save the results of detection, segmentation, and annotation to the local temporary database. The button “Export” is to export the information from the database into a word file. The detected moles are enumerated in the text box in the below part so that the user may click to choose each detected mole.
  Step 2. Choose an image to analyze, as shown in Figure 2(b). The user may click the button “Input an Image” to load an image. Or the user may load all the images in a specified file folder, by clicking the button “Choose a Folder.” After loading all the images files in the supported formats, the user may choose an image file by clicking the file name in the file list box in the left region of DiaMole.
  Step 3. Detect and segment the moles in the given image, as shown in Figure 3. The bounding boxes of the moles in the given images may be detected using four algorithms, that is, YOLOv3, RetinaNet, FR-CNN, and ALL. Click the button to choose the object detection algorithm. There is only one mole segmentation algorithm UNet, and the mole in each bounding box is automatically segmented.
  The visualization region under the four buttons has three pages, that is, “raw,” “detect,” and “draw.” The page “raw” gives the original image. The bounding boxes and the masks of the detected moles are illustrated in the page “detect.” The detected moles are listed in the below part of the right region. The page “draw” gives the canvas for the user to draw a bounding box to cover a user-detected candidate mole.
  Step 4. Define a bounding box for a candidate mole missed by DiaMole, as shown in Figure 4. Firstly, the user may switch to the page “draw” in the middle region of DiaMole, as shown in Figure 4(a). The user may then use the mouse to draw a rectangle to cover a candidate mole in the image, as shown in Figure 4(b). DiaMole asks whether the user wants to save this rectangle as a candidate mole. The user may click “Yes,” if satisfied with the drawn bounding box. Otherwise, the user may just click “No” to cancel this draw bounding box. The newly drawn bounding box is shown in the image after the user clicks “Yes,” as shown in Figure 4(c). The user can annotate a candidate mole with any text after clicking the mole's name in the right region of DiaMole, as shown in Figure 4(d).
  Step 5. Click the button “Save” in the right region of DiaMole to save the current data. The masks and annotations of all the candidate moles will be saved into the local database.
  Step 6. Click the button “Export” in the right region of DiaMole to export the current data. The masks and annotations of all the candidate moles will be exported as an annotation report, and the data may be analyzed by other tools.
  Step 7. Click the button “Help” in the left region of DiaMole to get the instruction. The usage instruction of DiaMole will be popped up if you click the “Help” button.

### 3.3. Performance Evaluation of Mole Detection Algorithms

DiaMole used three popular object detection algorithms to detect the two types of objects in the MoleMapper dataset. The integration algorithm ALL used the NMS strategy to combine the detection results of the above three algorithms. An object detection algorithm's performance is evaluated by mean average precision (mAP). The mAP is widely used in measuring the object detection algorithms [13, 15, 16]. In the detection of moles and coins, curves can be drawn for every class according to recall and precision. The average precision (AP) is the area under the corresponding curve, and mAP is the average AP of multiple targets. The higher the mAP is, the better the algorithm's performance is.

In this study, we used three object detection algorithms, YOLOv3, RetinaNet, and FR-CNN. We can get the positions of the coins and moles in the images by these algorithms. During the training phase of YOLOv3, we used the momentum to optimize the weights. The learning rate was 0.0001, and the cost function was optimized using 10705 epochs. When training the Faster R-CNN, we used the momentum to optimize the weights, set the learning rate to 0.0001, and used 150000 epochs to optimize the cost function. When training the RetinaNet, we used the momentum to optimize the weights, set the learning rate 0.0005, and used 150000 epochs to optimize the cost function.

The four algorithms were evaluated for their detection performances of the two classes “Coin” and “Mole,” as shown in Figure 5. This study randomly split the MoleMapper dataset into 70% training dataset and 30% test dataset. Both FR-CNN and RetinaNet performed very well on detecting the objects in the class “Coin” but only achieved 0.644 in AP for detecting moles. YOLOv3 did not perform well on detecting the moles. FR-CNN achieved the best mAP = 0.835. When we used NMS to integrate the above algorithms, the integration algorithm ALL achieved mAP = 0.4228. Although the integration performance was not good, ALL avoided missing the detection of moles by integrating the three object detection algorithms.

### 3.4. Demonstration of the Segmented Moles

This section demonstrated that object detection was necessary for detecting moles in the mobile phone images, as shown in Figure 6. The segmentation algorithm UNet did not find any moles in the mobile phone image, as shown in Figures 6(a) and 6(b). If the object detection algorithm ALL was used to find the bounding boxes of the candidate moles in the image, the UNet model accurately detected the two moles' precise boundaries from the mobile phone image.

### 3.5. Performance of DiaMole on the Locally Collected Dataset

The mole images from six other locally recruited participants were collected, and their information was summarized in Figure 7. These data were used to evaluate how DiaMole performed on the mobile phone images captured in everyday life, as shown in Figure 8. RetinaNet detected a light-colored mole, while the other two algorithms FR-CNN and YOLOv3 missed it, as shown in Figure 8(a). All three algorithms detected the right mole, but FR-CNN and RetinaNet recognized the scar as a mole, as shown in Figure 8(d). FR-CNN detected the mole correctly in Figures 8(c) and 8(e), but the other two algorithms missed. So overall FR-CNN may serve as a good mole detection algorithm. The user may also choose the integrated algorithm ALL or the other two algorithms.

### 3.6. Performance of DiaMole on Mole Images of Different Qualities

To verify the software's performance on mole images obtained using different mobile operating systems, this study took additional mole images by three different mobile phones for three participants, as shown in Figure 9. The mole images were obtained at different image qualities, and the mobile operating systems were iOS 14.2, Android 10, and Android 10.1.0, respectively. As Figure 9 illustrated, the mole images were taken by different mobile operating systems and had complicated backgrounds. But DiaMole detected all the eye-observable moles. So the image quality showed neglectable impacts on DiaMole's mole detection performance.

### 3.7. Evaluation of Each Algorithm's Running Time

This study used three object detection algorithms to detect the moles, and then the algorithm UNet was used to get the precise border of each detected mole's bounding box. In order to evaluate how fast each object detection algorithm ran on an image, this study chose the nine images from Figure 9 and ran YOLOv3, RetinaNet, and FR-CNN on each image. The average running time of each algorithm on each mobile operating system was illustrated in Figure 10. So FR-CNN ran the fastest to detect moles on the mobile-taken mole images, and it completed its task no more than 15.95 seconds for the mole images taken by both iOS and Android. YOLOv3 was the slowest mole detection algorithm. The data in the above sections suggested that a combined result of all the three algorithms (the mode “ALL”) may be chosen to avoid any missed moles.

## 4. Discussion

This study developed easy-to-use integrated software, DiaMole, to help dermatological researchers collect and annotate the moles in the mobile phone-captured images. Three popular object detection algorithms YOLOv3, FR-CNN, and RetinaNet were integrated to find the bounding boxes of candidate moles. Their results may be further integrated using the NMS strategy. The candidate mole in a given bounding box will be automatically segmented using the UNet model. The users may manually draw a bounding box to cover a mole missed by DiaMole and annotate these candidate moles based on their experiences.

All the detected moles and their annotations may be exported for further investigations.

## 5. Conclusions

The proposed software DiaMole may help the dermatological researchers investigate the moles in mobile phone-captured images. Melanoma is a major lethal skin cancer, and its early diagnosis will greatly increase the survival rate of the patients. Melanoma may develop from moles, but the patients may ignore the changes of moles in many cases. This study demonstrated that the previous mole or melanoma detection algorithms were usually trained over the dermoscopic images and did not perform well on the mobile phone-captured skin images. DiaMole utilized the object detection algorithms to ensure that the segmentation algorithm was not distracted from the background objects. But the DiaMole's running time is a little long, and this will affect the users' efficiency. In future studies, we plan to test and integrate more lightweight neural network models into DiaMole. The neural network Python libraries with support for parallel computing will be preferred to reduce the detection time.

## Figures and Tables

**Figure 1:** Workflow of DiaMole. Moles in the input images were detected by the algorithms YOLOv3, FR-CNN, RetinaNet, and ALL. After that, each bounding box was cropped out and segmented by the UNet. The users may annotate these moles. The annotation information and the mask images of the detected moles will be assembled as the final mole report.

**Figure 2:** Graphical user interface (GUI) of DiaMole. (a) After running the software, DiaMole's GUI is shown above. (b) An image is loaded into the GUI.

**Figure 3:** Mole detection and segmentation. After running the object detection algorithm, the detection result and the mask label result are shown in the software.

**Figure 4:** Draw the bounding box for a candidate mole. (a) The user may draw a rectangle as the bounding box for a candidate mole missed by DiaMole. (b) DiaMole lets the user decide whether the rectangle is good enough for the candidate mole. (c) The user-defined bounding box is shown in the image, and its name is listed in the right region. (d) Click a bounding box name in the right region to annotate it.

**Figure 5:** Performances of the four object detection algorithms. The column series AP (Coin) and AP (Mole) gave the averaged precision (AP) for the two classes of objects “Coin” and “Mole,” and the column series mAP gave the mean averaged precision (mAP) for the two classes.

**Figure 6:** Segmenting moles from a mobile phone image of the locally collected sample male-4. (a) The original mobile phone image. (b) UNet-segmented mask on the original image. (c) UNet-segmented mask on the bounding boxes from the object detection algorithm ALL.

**Figure 7:** Summary of the 7 locally collected samples using iPhone 6S. The samples are annotated with the gender and age information.

**Figure 8:** Detection of the moles in the mobile phone images of the six locally recruited participants. (a) Female-1, (b) female-2, (c) female-3, (d) male-1, (e) male-2, and (f) male-3.

**Figure 9:** Detection of the moles obtained using different mobile operating systems. (a) iOS 14.2, (b) Android 10, and (c) Android 10.1.0.

**Figure 10:** Running time of the three mole detection algorithms. The horizontal axis gave the algorithm names. The vertical axis gave the running time of each algorithm on each mobile operating system. Three participants were tested, and the running time was averaged over the three images taken by each mobile operating system.

## Data Availability

The program and the phone-captured mole images of seven local participants are available at http://www.healthinformaticslab.org/supp/.
